The article "Morusin alleviates mycoplasma pneumonia via the inhibition of Wnt/β-catenin and NF-κB signaling" was published in 2019. Journal: Biosci Rep.

# Morusin alleviates mycoplasma pneumonia via the inhibition of Wnt/β-catenin and NF-κB signaling

**DOI:** 10.1042/BSR20190190

**Published:** 2019-06-20

**Authors:** Cunrong Chen, Jingjing Wang, Jianfei Chen, Lili Zhou, Hui Wang, Junnian Chen, Zhihui Xu, Shuaijun Zhu, Wei Liu, Ranjie Yu, Junli Lu, Haoteng Luo, Min Chen, Weiwen Chen

**Affiliations:** 1 Department of ICU, Fujian Medical University Union Hospital, Fuzhou, Fujian 350001, China; 2 Department of ICU, The Affiliated Hospital of Putian College, Putian, Fujian 351100, China; 3 Department of ICU, First Hospital of Quanzhou Affiliated to Fujian Medical University, Quanzhou, Fujian 362000, China

**Keywords:** Morusin, mycoplasma pneumonia, mice, NF-κB, Wnt/β-catenin

## Abstract

Morusin has been traditionally used for the treatment of *Mycoplasma pneumoniae* pneumonia (MPP), but the underlying mechanism remains elusive. The present study aimed to explore the mechanism by which morusin achieves efficacy on mycoplasma pneumonia. Mycoplasma pneumonia model was established in BALB/c mouse and the effects of morusin were evaluated in the model. Compared with the model group, DNA amount of *M. pneumoniae* decreased by 24.6 ± 3.14% and 47.6 ± 6.78% in low morusin (20 mg/kg) and high morusin (50 mg/kg) groups, respectively (*P*<0.05). Moreover, morusin treatment led to decreased levels of pro-inflammatory cytokines such as interleukin (IL)-6, IL-1β, and tumor necrosis factor α and increased level of anti-inflammatory IL-10 in mice lung tissue. Furthermore, morusin treatment inhibited the activation of Wnt/β-catenin and NF-κB pathways in mice lung tissue. Taken together, our results suggest that morusin relieves mycoplasma pneumonia via the inhibition of the activation of Wnt/β-catenin and NF-κB pathways, and is a potential natural agent for the treatment of mycoplasma pneumonia.

## Introduction

*Mycoplasma pneumoniae* pneumonia (MPP) is a common type of acquired pneumonia caused by *M. pneumonia* infection and is one of three most serious pediatric diseases worldwide [1]. Recently, *M. pneumoniae* became more resistant to the antibiotics, resulting in increased incidence of MPP and making the disease hard to cure and easy to recur. Furthermore, MPP could cause severe complications, such as asthma and pulmonary fibrosis, and the patients with MPP require intense care [2]. Therefore, it is urgent to develop effective treatments for MPP.

Cortex Mori (CM), the root bark of *Morus alba* L., is a commonly used drug in Chinese medicine. Several compounds have been isolated from CM including polyhydroxylated alkaloids, flavonoids, and stilbenoids [3,4]. Morusin is one of the major active substances isolated from CM that exhibits anti-tumor, anti-inflammation, and anti-fungal activities [5,6]. Morusin has been traditionally used for the treatment of MPP, but the underlying mechanism remains elusive. Morusin has been reported to induce apoptosis and inhibit NF-κB signaling in human cervical, liver, and colorectal carcinoma cells [7,8]. Therefore, we hypothesized that morusin may exhibit efficacy on MPP via inhibiting NF-κB signaling. The present study aimed to test this hypothesis. We established *M. pneumoniae* infected BALB/c mouse model of MPP, evaluated protective effects of morusin on MPP, and investigated the underlying mechanism.

The article "Morusin alleviates mycoplasma pneumonia via the inhibition of Wnt/β-catenin and NF-κB signaling" was published in 2019. Journal: Biosci Rep.

## Methods

### Animals

The present study was approved by Fujian Medical University Committee of Animal Care and Use and performed at Fujian Medical University Lab Animal Center. BALB/c mice (3-week old, 15 ± 1 g weight) were purchased from Fujian Medical University Lab Animal Center (Fuzhou, China) and kept in specific pathogen free (SPF) environment with free access to food and water. All mice were divided randomly into five groups (*n*=5) as control, model, azithromycin (AZM), low morusin (20 mg/kg), and high morusin (50 mg/kg). Morusin was isolated from the chloroform extract of *M. alba* root bark as described previously [9]. Mice in control group were treated with 100 μl normal saline by nasal drops, while mice in other groups were given nasal drops containing 100 μl *M. pneumoniae* suspension (1 × 10^7^ cu/ml) for 3 days. In addition, AZM, morusin (20 mg/kg), and morusin (50 mg/kg) groups were given 46.25 mg/g AZM (Pfizer, New York, U.S.A.), 20 mg/kg morusin, and 50 mg/kg morusin by gavage once at 10 am each day for 7 consecutive days, respectively. On day 7, all five mice in each group were killed by ether anesthesia for lung index calculation. Then, the lungs were harvested and dissected for further analysis.

### Histological analysis

Inferior lobe of the right lung was fixed with 4% paraformaldehyde, embedded with paraffin, and cut into series of sections. The sections were hydrated with xylene and alcohol, and then stained by hematoxylin and eosin (HE). The sections were then washed thoroughly and mounted for observation under optical microscope

### Polymerase chain reaction (PCR)

Lung tissues were harvested, homogenized, and resuspended in DNA extract buffer and boiled for 10 min, the mixture was then centrifuged at 12000 rpm for 5 min at 4°C. The supernatant was taken as the template for PCR using primers against 16S-rRNA (upstream 5′-GAATCAAAGTTGAAAGGACCTGC-3′ and downstream 5′-CTCTAGCCATTACCTGCTAAAGTC-3′, product size 266 bp) with the following conditions: initial denaturation at 94°C for 1 min, followed by 30 cycles of 94°C for 1 min, and 55°C for 1 min. The results were shown as Log (MP-NDA+1).

The article "Morusin alleviates mycoplasma pneumonia via the inhibition of Wnt/β-catenin and NF-κB signaling" was published in 2019. Journal: Biosci Rep.

### Enzyme-linked immunosorbent assay (ELISA)

Lung tissues were harvested, homogenized, and levels of interleukin (IL)-6, IL-1β, IL-10, and tumor necrosis factor α (TNFα) in lung tissues were measured using enzyme immunoassay kits (R&D systems, Minneapolis, MN, U.S.A.) according to the manufacturer’s instructions.

### Western blot analysis

Lung tissues were harvested and washed twice with PBS and lysed in ice-cold radio immunoprecipitation assay buffer (RIPA, Beyotime, Shanghai, China) supplemented with protease inhibitor cocktail (Sigma, St. Louis, MO, U.S.A.). Tissue lysates were centrifuged at 13000 rpm for 10 min at 4°C. The supernatant (20–30 μg of protein) was run on 10% SDS–PAGE gel and transferred onto polyvinylidene fluoride membranes (Millipore, Bredford, U.S.A.). The membranes were blocked with 5% skim milk, followed by incubation with primary antibodies against NF-κB, β-catenin, β-actin, and H3 (all from Santa Cruz Biotech, Santa Cruz, CA, U.S.A.) at 4°C overnight. The membranes were then washed with tris buffered saline with Tween 20 (TBST) and incubated with horseradish peroxidase conjugated secondary antibodies (Beyotime, Shanghai, China) at 37°C for 1 h. The membranes were then washed with TBST and visualized using enhanced chemiluminescence (ECL, Millipore).

### Statistical analysis

Data were presented as mean ± SD and analyzed using SPSS 18.0 software. Data for multiple comparisons were performed by one-way ANOVA followed by Dunnett’s test. A value of *P*<0.05 was considered statistically significant.

## Results

### Morusin relieved *M. pneumoniae* induced inflammatory damage of lung tissues

HE staining of mice lung tissues showed that lung structure was normal without any obvious lesion in bronchial tube pulmonary alveo in control mice (Figure 1A). In *M. pneumoniae* infected mice, the alveolar walls were thickened, and narrowed bronchial tubes as well as capillary blood congestion, were observed (Figure 1B). In AZM and morusin-treated mice, no obvious inflammation infiltration was observed in the bronchus. Only a small amount of blood vessels exhibited mild expansion hyperemia and few bronchial tubes were narrowed (Figure 1C–E). These observations indicate that morusin could relieve inflammatory lung tissue damage after *M. pneumoniae* infection.

**Figure 1:** Histological analysis of mouse lung tissues in each group HE staining. Scale bar: 20 μm.

### Morusin reduced *M. pneumoniae* load in infected mice

Next we determined DNA amount of *M. pneumoniae* in the five groups of mice. PCR analysis showed that DNA amount of *M. pneumoniae* in model mice was the highest among all groups. Compared with the model mice, DNA amount of *M. pneumoniae* decreased by 32.7 ± 4.89%, 24.6 ± 3.14%, and 47.6 ± 6.78% in AZM, morusin (20 mg/kg), and morusin (50 mg/kg) groups, respectively (Figure 2, *P*<0.05).

The article "Morusin alleviates mycoplasma pneumonia via the inhibition of Wnt/β-catenin and NF-κB signaling" was published in 2019. Journal: Biosci Rep.

**Figure 2:** DNA amount of *Mycoplasma pneumoniae* in mouse lung tissues in each group DNA amount of *M. pneumoniae* was measured by PCR. Data were presented as mean ± SD, compared with model group, *P < 0.05, **P < 0.01; n = 5.

### Morusin inhibited pro-inflammatory cytokine production in *M. pneumoniae*-infected mice

Inflammatory cytokines play an important role in inflammatory response. We wondered whether morusin could regulate cytokine levels such as IL-6, IL-10, IL-1β, and TNF-α after *M. pneumoniae* infection. ELISA assay showed that IL-6, IL-1β, and TNF-α levels in mice lung tissues significantly increased in the model mice compared with control mice, but reduced to normal levels after AZM or morusin treatment (Figure 3A–C, *P*<0.05). On the other hand, the level of IL-10 significantly decreased in *M. pneumonia*-infected mice lung tissues (*P*<0.05), which was partially restored by AZM or morusin treatment (Figure 3D).

**Figure 3:** Effects of morusin on cytokine levels in mouse lung tissues in each group *M. pneumoniae*-induced mice were treated with AZM and morusin (20, 50 mg/kg), levels of IL-6 (**A**), IL-1β (**B**), TNF-α (**C**), and IL-10 (**D**) were determined by ELISA. Data were presented as mean ± SD, compared with control group, ^##^*P*<0.01; compared with model group, *P<0.05, **P<0.01; *n*=5.

### Morusin inhibited Wnt/β-catenin and NF-κB signaling

Wnt/β-catenin and NF-κB signaling pathways play a critical role in the regulation of inflammatory response [10,11]. Therefore, we examined the effects of morusin on β-catenin and NF-κB p65 levels. Western blot analysis showed that the levels of β-catenin and NF-κB p65 increased significantly in the model mice compared with control mice (Figure 4A–D, *P*<0.05). However, AZM or morusin treatment significantly decreased the levels of β-catenin and NF-κB p65 in mice lung tissue compared with model mice (*P*<0.05).

**Figure 4:** Effects of morusin on β-catenin and NF-κB p65 level in mouse lung tissues in each group β-catenin (**A,B**) and NF-κB p65 (**C,D**) were detected by Western blot analysis. β-actin and H3 were used as loading control. Data were presented as mean ± SD, compared with control group, ^##^*P*<0.01; compared with model group, **P<0.01; *n*=5.

## Discussion

With the increasing morbidity of MPP and the resistance to macrolides antibiotics [12], the incidences of severe MPP and extrapulmonary complications have increased substantially. MPP and the extrapulmonary complications result in multiple organ failure and even death. In the present study, we demonstrated the efficacy of morusin in *M. pneumoniae*-infected BALB/c mice.

The article "Morusin alleviates mycoplasma pneumonia via the inhibition of Wnt/β-catenin and NF-κB signaling" was published in 2019. Journal: Biosci Rep.

We found that treatment with AZM and morusin significantly alleviated inflammatory response in *M. pneumoniae*-infected mice. IL-6, TNF-α, IL-1β, and IL-10 are important cytokines involved in regulating inflammatory response. IL-6 is generated in Th2 cells, fibroblast cells and macrophages, and is a key pro-inflammatory cytokine to promote inflammatory response. IL-6 level was increased in children infected with community-acquired pneumonia [13]. TNF-α and IL-1β are released in the early stage of inflammatory response, and they increase the permeability of vascular endothelial cells and promote the synthesis and release of other cytokines [14]. IL-10 is synthesized in Th2 cell and mononuclear macrophage, and inhibits the generation and release of IL-2 and IFN-γ by Th1 cells to suppress immune response. Our study showed that morusin treatment could reduce the release of pro-inflammatory cytokines IL-6, TNF-α, and IL-1β while increasing the production of anti-inflammatory cytokine IL-10 [15].

Wnt/β-catenin signaling is implicated in a variety of diseases including cancer and inflammation [16,17]. Previous studies reported that NF-κB pathway plays a crucial role in regulating inflammation response in the lung tissues [18,19]. Cytokines such as TNF-α, IL-1β, IL-8, and IL-6 can induce NF-κB overexpression [20]. In the present study, we found that morusin significantly inhibited the expression of β-catenin and NF-κB p65, which is the active form of NF-κB. Notably, it was recently reported that morusin inhibited RANTES/CCL5 and TARC/CCL17 secretion via the suppression of NF-κB p65 phosphorylation in TNF-α and IFN-γ-stimulated HaCaT keratinocytes [21]. Therefore, Morusin may serve as a potential anti-inflammatory agent by acting as an inhibitor of Wnt/β-catenin and NF-κB pathways. Further studies are needed to investigate how morusin modulates NF-κB p65 phosphorylation.

In summary, our results suggest that morusin is a natural product that effectively relieves *M. pneumoniae*-induced inflammation in mice lung tissue, decrease *M. pneumonia* load, inhibit the generation of inflammatory cytokine, and suppress the activation of Wnt/β-catenin and NF-κB pathways. Morusin is a potentially new natural agent for the treatment of mycoplasma pneumonia.

## Abbreviations

AZM: azithromycin
CM: Cortex Mori
HE: hematoxylin and eosin
IL: interlukin
MPP: *Mycoplasma pneumoniae* pneumonia
TBST: tris buffered saline with Tween 20
TNFα: tumor necrosis factor α

The article "Morusin alleviates mycoplasma pneumonia via the inhibition of Wnt/β-catenin and NF-κB signaling" was published in 2019. Journal: Biosci Rep.

## References

[1] FerrerB.E., WebsterJ., BruceJ., Narh-BanaS.A., NarhC.T., AlloteyN.K. (2016) Integrated community case management and community-based health planning and services: a cross sectional study on the effectiveness of the national implementation for the treatment of malaria, diarrhoea and pneumonia. Malar. J.15, 34010.1186/s12936-016-1380-927371259PMC4930600

[2] WoodP.R., KampschmidtJ.C., DubeP.H., CagleM.P., ChaparroP., KetchumN.S. (2017) Mycoplasma pneumoniae and health outcomes in children with asthma. Ann. Allergy Asthma Immunol.119, 146–15210.1016/j.anai.2017.05.02228634021PMC5590634

[3] ParkJ.H., JungY.J., JungJ.W., ShresthaS., HanD., LimD.W. (2015) Two new isoarylbenzofuran diglucosides from the root bark of Morus alba. J. Asian Nat. Prod. Res.17, 357–36310.1080/10286020.2014.97177525401999

[4] LiangJ.H., FuY.W., ZhangQ.Z., XuD.H., WangB. and LinD.J. (2015) Identification and effect of two flavonoids from root bark of Morus alba against Ichthyophthirius multifiliis in grass carp. J. Agric. Food Chem.63, 1452–145910.1021/jf505544e25603693

[5] de SouzaM.M., BittarM., Cechinel-FilhoV., YunesR.A., MessanaI., Delle MonacheF. (2000) Antinociceptive properties of morusin, a prenylflavonoid isolated from Morus nigra root bark. Z. Naturforsch. C.55, 256–26010.1515/znc-2000-3-41810817216

[6] LeeJ.C., WonS.J., ChaoC.L., WuF.L., LiuH.S., LingP. (2008) Morusin induces apoptosis and suppresses NF-kappaB activity in human colorectal cancer HT-29 cells. Biochem. Biophys. Res. Commun.372, 236–24210.1016/j.bbrc.2008.05.02318485277

[7] LimS.L., ParkS.Y., KangS., ParkD., KimS.H., UmJ.Y. (2014) Morusin induces cell death through inactivating STAT3 signaling in prostate cancer cells. Am. J. Cancer Res.5, 289–29925628938PMC4300697

[8] WangL., GuoH., YangL., DongL., LinC., ZhangJ. (2013) Morusin inhibits human cervical cancer stem cell growth and migration through attenuation of NF-kappaB activity and apoptosis induction. Mol. Cell. Biochem.379, 7–1810.1007/s11010-013-1621-y23543150

[9] VochyánováZ., PokornáM., RotreklD., SmékalV., FictumP., SuchýP. (2017) Prenylated flavonoid morusin protects against TNBS-induced colitis in rats. PLoS ONE12, e018246410.1371/journal.pone.018246428797051PMC5552281

[10] LiB., ZengM., HeW., HuangX., LuoL., ZhangH. (2015) Ghrelin protects alveolar macrophages against lipopolysaccharide-induced apoptosis through growth hormone secretagogue receptor 1a-dependent c-Jun N-terminal kinase and Wnt/beta-catenin signaling and suppresses lung inflammation. Endocrinology156, 203–21710.1210/en.2014-153925337654

[11] GuoL., WangT., WuY., YuanZ., DongJ., LiX. (2016) WNT/beta-catenin signaling regulates cigarette smoke-induced airway inflammation via the PPARdelta/p38 pathway. Lab. Invest.96, 218–22910.1038/labinvest.2015.10126322419

The article "Morusin alleviates mycoplasma pneumonia via the inhibition of Wnt/β-catenin and NF-κB signaling" was published in 2019. Journal: Biosci Rep.

[12] WangH. and HeH. (2018) Characterization of multidrug-resistant Klebsiella pneumoniae isolated from the Chinese cobra Naja atra in a Beijing suburb. Biocell42, 47–5410.32604/biocell.2018.07006

[13] OdehA.N. and SimeckaJ.W. (2016) Regulatory CD4+CD25+ T cells dampen inflammatory disease in murine mycoplasma pneumonia and promote IL-17 and IFN-gamma responses. PLoS ONE11, e15564810.1371/journal.pone.0155648PMC486668027175511

[14] JiangY.H., YuJ.E., GuoA.H., LiX., LinY., JiangZ.Y. (2016) Ameliorative effects of Qingfei Tongluo formula on experimental mycoplasmal pneumonia in mice. J. Nat. Med.70, 145–15110.1007/s11418-015-0944-226590157

[15] ChenH., LiN., WanH., ChengQ., ShiG. and FengY. (2015) Associations of three well-characterized polymorphisms in the IL-6 and IL-10 genes with pneumonia: a meta-analysis. Sci. Rep.5, 855910.1038/srep0855925708204PMC4338428

[16] BastakotyD. and YoungP.P. (2016) Wnt/beta-catenin pathway in tissue injury: roles in pathology and therapeutic opportunities for regeneration. FASEB J.30, 3271–328410.1096/fj.201600502R27335371PMC5024694

[17] TianH., CongP., QiR., GaoX., LiuX., LiuH. (2017) Decreased invasion ability of hypotaurine synthesis deficient glioma cells was partially due to hypomethylation of Wnt5a promoter. Biocell41, 27–32

[18] ChenL., YanX., YanQ., FanJ., HuangH., ShiX. (2015) The modified JiuWei QiangHuo decoction alleviated severe lung injury induced by H1N1 influenza virus by regulating the NF- kappa B pathway in mice. Evid. Based Complement. Alternat. Med.2015, 7907392608994710.1155/2015/790739PMC4451524

[19] CyphertT.J., MorrisR.T., HouseL.M., BarnesT.M., OteroY.F., BarhamW.J. (2015) NF-kappaB-dependent airway inflammation triggers systemic insulin resistance. Am. J. Physiol. Regul. Integr. Comp. Physiol.309, R1144–R115210.1152/ajpregu.00442.201426377563PMC4666958

[20] PintoR., HeroldS., CakarovaL., HoegnerK., LohmeyerJ., PlanzO. (2011) Inhibition of influenza virus-induced NF-kappaB and Raf/MEK/ERK activation can reduce both virus titers and cytokine expression simultaneously in vitro and in vivo. Antiviral Res.92, 45–5610.1016/j.antiviral.2011.05.00921641936

[21] JinS.E., HaH., ShinH.K. and SeoC.S. (2019) Anti-allergic and anti-inflammatory effects of Kuwanon G and Morusin on MC/9 mast cells and HaCaT keratinocytes. Molecules24, pii: E26510.3390/molecules24020265PMC635950530642008

